The article "Tea Drinking and the Risk of Carcinoma of the Urinary Bladder: A Meta-Analysis" was retracted in 2023. Reasons: signs of a paper mill; compromised peer review; unreliable results or conclusions.

# Tea Drinking and the Risk of Carcinoma of the Urinary Bladder: A Meta-Analysis

**DOI:** 10.1155/2023/2891120

**Published:** 2023-04-07

**Authors:** Qier Xia, Jun Li, Yifan Shen, Dahong Zhang

**Affiliations:** ^1^Suzhou Medical College of Soochow University, Soochow 215000, China; ^2^Department of Urology, Zhejiang Provincial People's Hospital, People's Hospital of Hangzhou Medical College, No. 158, Shangtang Road, Xiacheng District, Hangzhou 310014, Zhejiang, China; ^3^Department of Urology, Pudong New Area People's Hospital, Shanghai 201299, China

## Abstract

**Objective:**

For evaluation of the correlation between tea drinking and the risk of carcinoma of the urinary bladder.

**Methods:**

By searching PubMed, Embase, and Cochrane Library databases, the original studies on tea drinking and carcinoma of the urinary bladder risk were collected, the data were extracted, and meta-analysis package 5.2-0 of R language was used for meta-analysis.

**Results:**

This study contained 11 researches, composed of 7686 patients and 10320 controls. Tea drinking was not linked to carcinoma of the urinary bladder risk (OR:1.02, 95%CI: 0.95–1.11).

**Conclusion:**

Tea drinking may not be linked to carcinoma of the urinary bladder, but more definitive results are needed from higher-quality trials.

## 1. Introduction

Carcinoma of the urinary bladder is the most frequently diagnosed tumor in the urinary system, ranking 11th in the incidence of malignant tumors. The annual number of carcinoma of the urinary bladder deaths is about 170,000 [1]. According to the paper published by Lu Xin et al., the number of carcinoma of the urinary bladder deaths in China from the past ten years was 37,237, and the proportion of carcinoma of the urinary bladder deaths increased from 1.01% in 2004 to 1.23% in 2018 [2]. Bladder cancer can be divided into nonmuscule invasive bladder cancer (NMIBC) and muscule invasive bladder cancer (MIBC). At present, the preferred treatment for NMIBC is transurethral resection of bladder tumor (TURBT) plus postoperative adjuvant intravesical perfusion (chemotherapy and immunotherapy). The preferred treatment for MIBC is radical cystectomy plus pelvic lymph nodes. TURBT not only has a diagnostic role but also has a therapeutic effect, according to the pathological characteristics of the tumor for radical treatment.

Although the exact risk elements for carcinoma of the urinary bladder have not been elucidated, studies have found that there are risk elements linked to carcinoma of the urinary bladder. Various geographical factors, genes, and personal habits are Risk elements for carcinoma of the urinary bladder, such as smoking, age, etc. [3–5]. Vegetables and fruits can lower carcinoma of the urinary bladder risk [6, 7]. Some drugs even affect the risk of carcinoma of the urinary bladder. For example, the drug insulin may increase carcinoma of the urinary bladder risking smokers [8], but nonsteroidal anti-inflammatory drugs excluding aspirin can lower carcinoma of the urinary bladder risking nonsmokers [9, 10]. Tea drinking is a popular beverage all over the world and continuous studies have found its medical and health care effects. Current studies have found that tea can not only lower the risk of cardiovascular and cerebrovascular diseases [11, 12], but also lower the risk of oral cancer [13]. Although some studies have assessed the connection between tea drinking and carcinoma of the urinary bladder, the results are inconsistent [14–16]. Hence, this study mainly used meta-analysis to explore whether tea drinking is a hazard element for carcinoma of the urinary bladder.

## 2. Data and Methods

### 2.1. Inclusion Criteria and Exclusion Criteria Inclusion Criteria

Inclusion criteria is as follows: (1) Human subjects; (2) the article type was case-control study; and (3) the language is English. Exclusion criteria is as follows: (1) Review, abstracts, and conference papers; (2) unable to obtain the full text; (3) low-quality literature (NOS ≤ 5 points); (4) human in vitro test, (5) concomitant with other cancers; and (6) metastatic bladder cancer.

### 2.2. Literature Retrieval

“Carcinoma of the urinary bladder,” “bladder carcinoma,” “bladder neoplasm,” and “tea” were used as keywords to search the databases (PubMed, Embase, and Cochrane Library) for articles published before May 2022 that met the inclusion exclusion criteria.

### 2.3. Literature Screening and Data Extraction

Two investigators independently conducted literature search and performed literature screening based on inclusion and exclusion criteria, with confirmation by the principal investigator in case of disagreement. Data extraction was performed separately for the included literature by developing data collection forms including authors, follow-up time, sample size, and RR or OR including 95% CI for carcinoma of the urinary bladder as well as nontumor control group. If the article examined the effect of different tea drinking on carcinoma of the urinary bladder development, the minimum amount of data was extracted.

### 2.4. Evaluation of Literature Quality

Two investigators independently evaluated the quality of literature using the Newcastle-Ottawa Scale (NOS), and in case of disagreement, the primary investigator confirmed the quality. The scale was scored out of 9, and articles with a score of ≥7 were regarded as high quality, and articles with a score of >6 were included in the study.

### 2.5. Statistical Analysis Methods

The meta-analysis package of R language 4.1.0 software was used for data analysis. OR or RR values with 95% CI were used to describe the link between tea drinking and the risk of carcinoma of the urinary bladder. *I*^2^ values were used to quantify the heterogeneity of the study for analysis, with *I*^2^ < 50% indicating moderate heterogeneity and selection of a fixed-effects model and *I*^2^ ≥ 50% represents high levels of heterogeneity. *I*^2^ ≥ 50%, sensitivity analysis was performed one-by-one. Sensitivity analysis was performed to discover the origin of heterogeneity and the robustness of the data results. Egger's test was used to quantify publication bias and was considered statistically significant at *p* < 0.05, meaning that publication bias was present. Funnel plots were drawn and the distribution characteristics were observed to examine the publication bias of the included literature.

## 3. Results

357 literature studies were searched in PubMed, Embase, and Cochrane Library databases by keywords, and 11 literature studies were finally included for analysis through inclusion and exclusion criteria. The specific screening process is shown in Figure 1.

The essential features of the incorporated studies are listed in Table 1.

Studies were conducted mainly in Western countries, with only one study conducted in China, and all included studies were retrospective studies using either questionnaires or a combination of questionnaires and interviews. 7,686 patients with carcinoma of the urinary bladder and 10,320 patients without cancer were included. Ten studies had NOS scores greater than 7, and they were considered high quality studies, and one study with a NOS score of 6 was considered lower quality but was still included in the analysis.

Eleven papers reported a link between tea drinking and the risk of carcinoma of the urinary bladder. The result of *I*^2^ was 62%, indicating a high heterogeneity in the included literature, and hence a random effects model was used for the analysis. The results of the meta-analysis showed an OR of 1.02 with 95% CI of 0.93–1.11. The forest plot is shown in Figure 2.

Publication bias can be observed through funnel plot, which is roughly symmetrical in this study (Figure 3). Publication bias was measured by Egger's test (*p* = 0.4651), so there was no publication bias (Figure 4).

Heterogeneity analysis was performed using one-by-one exclusion to discover the origin of heterogeneity, and the results showed that by removing one study at a time and then analyzing it, the findings were stable (Figure 5).

## 4. Discussion

Carcinoma of the urinary bladder is multicentric in nature and has a high recurrence rate after surgery, requiring frequent reviews and long-term follow-up, and is hence a great economic burden for the patient's family and society. The factors of carcinoma of the urinary bladder development have been a hot topic of research. The use of natural food components for human tumor prevention is a hot topic of international research. For example, vegetables and fruits can lower carcinoma of the urinary bladder risk [6, 7]. The medicinal health value of tea has been studied since ancient times. For example, the medicinal effects of tea were reported in the Compendium of Materia Medica. Scientists at home and abroad have conducted in-depth studies on the anticancer and cardiovascular protective effects of tea [11–13].

The results of the current anticancer experiments with tea in animals are encouraging. Green and mixed teas inhibited dimethylbenzanthracene (DMBA) induced oral cancer in golden gopher [28]; green and black teas inhibited esophageal carcinogenesis by blocking the synthesis of methylbenzylnitrosamine (NMBzA) precursors in rats [29]. The main active ingredient in tea is tea polyphenol (Epigallocatechin-3-Gallate (EGCG)), which differs among different types of tea, for example, green tea polyphenol extract is catechin while black tea polyphenol extract is theaflavin. Tea polyphenols have excellent antitumor activity [30], and the main mechanisms involve antioxidant effects, immunomodulatory effects, inhibition of oncogene expression, induction of apoptosis, and prevention of DNA damage [31–34]. Although much in vitro evidence suggests that tea has good anticancer effects, real data studies on tea drinking against carcinoma of the urinary bladder are mainly retrospective case-controlled studies and prospective single cohort studies, usually using questionnaires, and there is a lack of high-quality randomized controlled placebo studies with large samples.

Al-Zalabani et al. showed in their article that a higher level of tea consumption was associated with lower risk of bladder cancer incidence. In addition, dose-response analyses showed a lower bladder cancer risk with increment of 100 ml of tea consumption per day [35].

In summary, the results of this paper suggest that tea drinking may not lower the risk of carcinoma of the urinary bladder, but there are still some limitations of this study, mainly in the following aspects: (1) All included literature are retrospective case-control studies, and there are no randomized, double-blind, placebo-controlled studies, which would lower the reliability of the data in this study. (2) Most of the included studies considered the connection between tea and carcinoma of the urinary bladder risking general, without considering the type of tea and the amount of tea consumed, which prevented a more precise analysis of this study. (3) As there were no subgroup analyses of age, gender, and other adverse lifestyle habits in the included literature, the corresponding data could not be obtained for analysis in this study. Hence, high-quality randomized controlled placebo studies with large samples are needed to confirm whether tea drinking lowers the risk of carcinoma of the urinary bladder.

## Figures and Tables

**Figure 1:** Literature screening process.

**Figure 2:** Forest map.

**Figure 3:** Funnel plot.

**Figure 4:** Egger's linear correlation diagram.

**Figure 5:** Sensitivity analysis.

**Table 1:** Basic features of included studies.

Authors	Follow-up time	Place	Patients with carcinoma of the urinary bladder	Nononcology patients	NOS
Lu et al. [17]	1996–1997	Taiwan	40	160	7
D'Avanzo et al. [18]	1985–1990	Italy	555	855	8
Clavel and Cordier [19]	1984–1987	France	690	690	8
Risch et al. [20]	1979–1982	Canada	835	792	7
Jensen et al. [21]	1979–1981	Denmark	388	787	7
Bianchi et al. [22]	1986–1989	United States	818	1297	8
Geoffroy-Perez et al. [23]	1984–1987	France	765	765	8
Woolcott et al. [24]	1992–1994	Canada	927	2118	8
De Stefani et al. [25]	1996–2000	Uruguay	255	501	6
Jiang et al. [26]	1987–1999	United States	1586	1586	8
Hemelt et al. [27]	2005–2008	China	827	769	6

## Data Availability

All data generated or analysed during this study are included in this published article.
